# Incidental Prostate Cancer at the Time of Cystectomy: The Incidence and Clinicopathological Features in Chinese Patients

**DOI:** 10.1371/journal.pone.0094490

**Published:** 2014-04-10

**Authors:** Jiahua Pan, Wei Xue, Jianjun Sha, Hu Yang, Fan Xu, Hanqing Xuan, Dong Li, Yiran Huang

**Affiliations:** Department of Urology, Renji Hospital, Affiliated to Shanghai Jiao Tong University, School of Medicine, Shanghai, China; University of British Columbia, Canada

## Abstract

**Objectives:**

To evaluate the incidence and the clinicopathological features of incidental prostate cancer detected in radical cystoprostatectomy (RCP) specimens in Chinese men and to estimate the oncological risk of prostate apex-sparing surgery for such patients.

**Methods:**

The clinical data and pathological feature of 504 patients who underwent RCP for bladder cancer from January 1999 to March 2013 were retrospectively reviewed. Whole mount serial section of the RCP specimens were cut transversely at 3–4 mm intervals and examined in same pathological institution.

**Results:**

Thirty-four out of 504 patients (6.8%) had incidental prostate cancer with a mean age of 70.3 years. 12 cases (35.2%) were diagnosed as significant disease. 4 cases were found to have apex involvement of adenocarcinoma of the prostate while in 5 cases the prostate stroma invasion by urothelial carcinoma were identified (one involved prostate apex). The mean follow-up time was 46.4±33.8 months. Biochemical recurrence occurred in 3 patients but no prostate cancer-related death during the follow-up. There was no statistical significance in cancer specific survival between the clinically significant and insignificant cancer group.

**Conclusions:**

The prevalence of incidental prostate cancer in RCP specimens in Chinese patients was remarkably lower than in western people. Most of the incidental prostate cancer was clinically insignificant and patient's prognosis was mainly related to the bladder cancer. Sparing the prostate apex was potentially associated with a 1.0% risk of leaving significant cancer of the prostate or urothelial carcinoma.

## Introduction

Bladder cancer is the second most common genitourinary malignancy worldwide and the most frequently diagnosed genitourinary cancer in China [1], [2]. It leads to significant morbidity and mortality. Up till now, RCP remains the golden standard for muscle invasive bladder cancer or recurrent superficial urothelial carcinoma at high risk [3]. Although the neobladder reconstruction and nerve-sparing technique offer a better quality of life for the patients, the recovery of erectile function and urinary continence after surgery are still far from satisfactory [4]. Therefore, the prostate apex-sparing or even the total prostate-sparing techniques have been developed to improve the postoperative urinary continence and sexual function [5], [6]. However, the potential risk of prostate cancer residue and prostatic involvement with urothelial carcinoma become a major concern for these techniques.

The incidence of prostate cancer varies significant among different countries and ethnic groups. It is quite frequently diagnosed in North America and Europe but rare in Asians [7]. According to the latest reports, the incidence rate was only 12.10/100 000 in China and 12.70/100 000 in Japan [2], [8]–[9]. More importantly, most of the prostate cancer diagnosed in the specimens from RCP for bladder cancer is considered as clinically insignificant disease [10]–[14]. However, in this issue, only few data of Chinese cohort are available with limited cases. In this study, we retrospectively reviewed 504 RCP cases for bladder cancer to investigate the incidence and clinicopathological features of incidental prostate cancer in RCP specimens in Chinese patients. To our knowledge, this study represents the largest series to date of incidental prostate cancer at RCP in China and even in Asia.

## Materials and Methods

### Cohort selection and pathological evaluation

The clinical data and pathological feature of 504 patients who underwent standard RCP for bladder cancer at our institution from January 1999 to March 2013 were retrospectively reviewed. As a tertiary referral center, these patients came from 31 out of 34 administrative zones of China. Patients with an abnormal result of digital rectal examination (DRE) or PSA suspicious of prostate cancer and finally confirmed by prostate biopsy before the surgery or patients having a history of prostate cancer were already excluded from the study. The study protocol was approved by the ethical committee of the faculty of medicine of Shanghai Jiao Tong University, School of Medicine. All patients enrolled in this study signed an informed consent before the surgery.

The preoperative assessment included DRE and upper urinary tract imaging such as intravenous urography (IVU), CT urography (CTU) or magnetic resonance urography (MRU). However, the PSA was only available in 296 cases before RCP. All the pathological examination was performed in the same institution. Whole mount serial section of the RCP specimens were cut transversely at 3–4 mm intervals. Besides the urothelial carcinoma of the urinary bladder, the location and tumor volume of the prostate cancer, prostate apex involvement, Gleason score, pathological staging and surgical margins were evaluated. Clinically significant prostate cancer was defined as a tumor volume≥0.5 ml; Gleason 4 or 5 pattern, extracapsular extension, seminal vesicle invasion, lymph node metastasis or positive surgical margins [15].

### Follow-up

The first postoperative PSA follow-up was scheduled at 3 months after the surgery, then every 3 months the first year, every 6 months the second year and annually thereafter. A biochemical recurrence was defined as an initial serum PSA of ≥0.2 ng/ml, with a second confirmatory level of PSA of >0.2 ng/ml [16].

### Statistical Analysis

Proportions of the variables were analyzed using Chi-square test or Fisher's exact test while mean values were compared with one-way ANOVA test. The cancer specific survival was described using Kaplan-Meier curves. Survival differences were compared by the Log-rank test. Statistical significance was set at P<0.05 and all the P values were two-sided. The SPSS 18.0 was applied to perform the data analysis.

## Results

### Incidental prostate cancer

In this study, 34 out of 504 patients (34/504, 6.8%) who underwent RCP had incidentally diagnosed prostate cancer. The mean age was 70.3±8.9 years and the mean follow-up was 46.4±33.8 months. A preoperative PSA was available in 23 cases with incidental prostate cancer and their median PSA was 2.67±2.24 ng/ml. A tumor volume of more than 0.5 cm^3^ was identified in 8 patients (8/34, 23.5%). 4 cases were found to have apex involvement of adenocarcinoma of the prostate while in 5 cases the prostate stroma invasion by urothelial carcinoma were identified (one involved the prostate apex). The detailed pathological staging and Gleason score were summarized in Table 1.

**Table 1:** Patients demographic data of incidental prostate cancer

	Incidental prostate cancer (n = 34)
Age at RCP (Year)	70.3±8.9 (range 52–86)
Follow-up (Months)	46.4±33.8 (range 1–135)
Significant prostate cancer	12 (35.2)
Pathological stage of prostate cancer	
pT2a	19 (55.9)
pT2b	9 (26.5)
pT2c	2 (5.9)
pT3a	3 (8.8)
pT3b	1 (2.9)
Gleason Score	
3	1 (2.9)
4	4 (11.8)
5	4 (11.8)
6	18 (52.9)
7	5 (14.7)
8	1 (2.9)
9	1 (2.9)
Prostate cancer volume ≥0.5 ml	8 (23.5)
Prostate cancer positive surgical margin	1 (2.9)
Prostate apex involvement by incidental prostate cancer	4(11.8)
Prostate stroma invasion by urothelial carcinoma	5 (14.7)

12 cases (12/34, 35.2%) were diagnosed as significant prostate cancer, while 22 (22/34, 64.8%) were clinically insignificant. The mean age of the patients with significant cancer and insignificant cancer was 66.83±6.83 years and 72.14±9.43 years, respectively. The preoperative PSA was available in 14 cases in insignificant cancer group with a median PSA of 2.0 ng/ml whereas available in 9 patients in significant cancer group with a median PSA of 3.7 ng/ml (P = 0.14). The positive surgical margin of prostate cancer was detected in 1 patient with significant disease. All the 4 cases with apex involvement of adenocarcinoma of the prostate were in significant cancer group and 3 of them had a preoperative PSA available. The median PSA of these 3 cases was 4.1 ng/ml. Although the prostate apex involvement was statistically higher in significant prostate cancer group, the biochemical recurrence rate was similar between the 2 groups during the follow-up. In addition, there was no statistical difference in pathological staging and the pelvic lymph node involvement of the bladder cancer between the 2 groups. The Clinical characteristics and pathologic feature of these 2 groups were listed in Table 2.

**Table 2:** Clinical data and pathological feature of significant and insignificant incidental prostate cancer

	Significant prostate cancer(%)	Insignificant prostate cancer(%)	P
Number of Cases	12	22	
Mean Age at RCP (Year)	66.83±6.83 (range 54–77)	72.14±9.43 (range 52–86)	0.096
Preoperative PSA(ng/ml)	2.0	3.7	0.141
Prostate apex involvement by prostate cancer	4 (33.3)	0 (0)	0.011
Prostate stroma invasion by urothelial carcinoma	3 (25.0)	2 (9.1)	0.319
Biochemical recurrence	2 (15.4)	1 (4.5)	0.234
Prostate cancer staging			
pT2a	1 (7.7)	18 (81.8)	
pT2b	5 (41.7)	4 (18.2)	
pT2c	2 (15.4)	0 (0)	
pT3a	3 (25.0)	0 (0)	
pT3b	1(7.7)	0 (0)	
Gleason Score			
3	0 (0)	1 (4.5)	
4	0 (0)	4 (18.2)	
5	0 (0)	4 (18.2)	
6	5 (41.7)	13 (59.1)	
7	5 (41.7)	0 (0)	
8	1 (7.7)	0 (0)	
9	1 (7.7)	0 (0)	
Bladder cancer staging			
pT1	1(8.3)	2(9.1)	0.614
pT2	5(41.7)	13(59.1)	
pT3	3(25.0)	5(22.7)	
pT4	3(25.0)	2(9.1)	
Bladder cancer lymph node involvement			
N0	10(83.3)	18(81.8)	0.742
N1	2(16.7)	3(13.6)	
N2	0(0)	1(4.5)	

### Prostatic stromal invasion by urothelial carcinoma

Prostatic stromal invasion is defined as the presence of invasive urothelial carcinoma nests or single cells penetrating through the basement membrane of prostatic ducts and acini. The prostate stroma invasion by bladder cancer were identified in 5 cases (one involved the prostate apex) in this cohort. 3 cases with prostate stroma invasion by urothelial carcinoma were in significant prostate cancer group while 2 in insignificant cancer group, respectively. (P = 0.32) When reviewing the pathological specimens, 4 out of these 5 cases were found to have high grade and multifocal urothelial carcinoma in urinary bladder and 3 of them had pelvic lymph node involvement.

### Biochemical recurrence and cancer specific survival

After RCP, the PSA was below the limit of detection in all cases. During the follow-up, biochemical recurrence occurred in 3 patients (3/34, 8.8%) without prostate apex involvement and then treated with androgen deprivation therapy.

As for the survival, 10 patients (10/34, 32.4%) died of metastatic bladder cancer, 3 in clinically significant prostate cancer group (3/12, 25.0%) and 7 in clinically insignificant group (7/22, 31.8%), whereas 1 (1/22, 4.5%) died of myocardial infarction. There was no prostate cancer-related death in both groups during the follow-up. Concerning the cancer specific survival between the clinically significant and clinically insignificant cancer group, there was no statistical significance identified. (P = 0.51) (Figure 1)

**Figure 1:** The Kaplan-Meier curves of cancer specific survival (including the urothelial carcinoma and the adenocarcinoma of the prostate) after radical cystoprostatectomy. The blue curve indicated the cancer specific survival of the cases with concomitant significant prostate cancer while the red curve showed the cancer specific survival of the cases with insignificant prostate cancer. There was no statistical significance identified between the 2 groups. (P = 0.51)

## Discussion

The frequency of incidental prostate cancer detected in RCP specimens is really variable all over the world. Abbas et al reported a 45% rate of incidental prostate cancer in a study of 40 cases [17]. Similar results were obtained by Montie et al, who found 33 of 84 men (33/84, 46%) undergoing cystoprostatectomy for bladder cancer had incidental prostate cancer [18]. However, the incidence rate was much lower in most of the Asian countries. According to the recent studies with 1207 cases from Asia, the prevalence of incidental prostate cancer was only about 10.9% [13], [19]–[25]. It was extremely low in China, Japan and India. Nevertheless, the incidental prostate cancer seemed to be rather frequent in Korea, which was similar to that of western countries. Base on the findings form Joung et al, the prevalence was as high as 50% [20]. (The incidence of incidental prostate cancer in Asian countries was summarized in Table 3.)

**Table 3:** The incidence of incidental prostate cancer in Asian countries

Nations	Authors	Samples	PCa Cases (%)	Clinical significance
Japan	Yumura et al [19]	59	3 (5.1)	N/A
Japan	Kurahashi et al [13]	251	31 (12.3)	9
Korea	Joung et al [20]	36	18 (50.0)	5
India	Desai et al [21]	44	3 (6.8)	N/A
Saudi	Mosli et al [22]	93	14 (15.1)	N/A
Iran	Hosseini et al [23]	50	7 (14.0)	4
China	Liu et al [24]	49	4 (8.2)	1
China	Zhu et al [25]	92	3 (3.3)	1
Present study	Pan et al	504	34 (6.8)	12
Overall		1207	132 (10.9)	

Such a significant discrepancy of prostate cancer prevalence between China or some other Asian countries and western countries might relate to genetic backgrounds, lifestyles, socioeconomical circumstances and dietary factors contributing to aggravate genomic susceptibility of prostate cancer. The varied geographic distribution across the world implies that the genetic background of prostate cancer might play a role in carcinogenesis. Carter et al reported that prostate cancer often occurred within a family [26]. In addition, males with a prostate cancer history in relatives of the first and second orders are more susceptible to have the disease. The twins studies demonstrated that monozygotic twins have a significantly increased risk than dizygotes in both brothers [27]–[28]. However, even though African Americans are highly susceptible to prostate cancer in United States, their original African nations actually have remarkably lower incidence [29]–[31], which suggests other important factors also influence the incidence of prostate cancer. Meanwhile, the significant difference of the lifestyle and dietary habits might also relate to prostate cancer incidence. Recent study revealed that the risk of prostate cancer was inversely associated with total dietary fiber intake, insoluble and legume fiber intakes, which are the staple diet in many Asian countries [32]. What's more, as the most popular drink in China and Japan, green tea might also contribute to reduce the prostate cancer risk. A study of Green tea and cancer prevention from Cochrane database demonstrated a decreased risk of prostate cancer in men consuming higher quantities green tea or green tea extracts [33]. Kim et al has also approved that the polyphenon E, a green tea extract was an effective chemopreventive agent in preventing the progression of prostate cancer to metastasis in TRAMP mice model [34].

Up till now, only few reports with limited cases of incidental prostate cancer prevalence in Chinese population are available. We retrospectively reviewed the clinical data and pathological features of 34 out of 504 RCP cases to evaluate the incidence of incidental prostate cancer and the prostate apex involvement in Chinese people.

In this study, incidental prostate cancer was found in 6.8% of RCP specimens, of which 35.2% were considered clinically significant. Patients with an abnormal result of DRE and finally diagnosed with prostate cancer before the surgery had been already excluded from the study. However, a PSA test was not routinely conducted in bladder cancer patients in our institution according to the PSA best practice policy of the American Urological Association, because most of the patients with muscle-invasive bladder cancer have a limited life expectancy whereas most prostate cancer has a relatively long nature history [35]. Thus, a routine PSA screen before RCP for muscle-invasive bladder cancer may only have limited value.

As for the pathological features of the incidental prostate cancer, we found that most of them was pT2a (19/34, 55.9%), with a Gleason score≤6 (27/34, 79.4%) suggesting a more favorable prognosis, which was similar to results of Muzzucchelli et al [12]. There were 3 patients developed a biochemical recurrence after the surgery whereas no patients died of prostate cancer during the follow-up period of this study. As Delongchamps et al mentioned, in patients with concomitant prostate cancer, the poor survival rate was due to the majority of advanced bladder tumors and the outcome would be probably similar as the patients without coexisting prostate cancer [36]. Other authors also have found the same results [17], [37]–[38]. In this case, another oncological problem would focus on whether incidental significant prostate cancer could affect the cancer specific survival of these patients. In this study, there are 12 cases with significant incidental prostate cancer and 22 cases with insignificant incidental prostate cancer. No statistic difference was found in mean age at cystoprostatectomy, in bladder cancer staging and in pelvic lymph node involvement rate by urothelial carcinoma between the groups. The Kaplan-Meier curves excluded a statistical difference in cancer specific survival rate between the 2 groups suggesting that the incidental significant prostate cancer also would not increase the risk of cancer specific mortality in patients with muscle-invasive bladder urothelial carcinoma.

RCP has traditionally been considered as a golden standard for the treatment of muscle-invasive bladder cancer [3]. However, the risk of erectile dysfunction and urinary incontinence following this procedure is considerable and might delay the patients' acceptance of RCP, which can adversely affect the prognosis of these patients. Considering the important role of prostate apex for urinary continence and the erectile function, the apex-sparing approach has become a treatment of choice for muscle-invasive bladder cancer. Davila et al. found that erectile function could be significantly preserved by prostate apex-sparing cystectomy [39], meanwhile Colombo et al also proved that after prostate apex-sparing cystectomy with orthotopic urinary diversion, daytime and nighttime continence could be immediate and complete after catheter removal with normal erectile function clinically documented [40]. However, the cancer control must be taken seriously when considering the quality-of–life. In our series, 5 cases (5/34, 14.7%) were found to have prostate-apex involvement by adenocarcinoma of the prostate or urothelial carcinoma. Since the incidence rate of incidental prostate cancer was 6.8% in RCP specimens and the prostate-apex involvement rate was 14.7% (4 apical involvement by incidental prostate cancer and 1 apical involvement by urothelial carcinoma), sparing the prostate apex would be potentially associated with a 1.0% risk of leaving significant cancer of the prostate or urothelial cancer, which was much lower than the estimated risk reported by Gakis et al from a Germany cohort [41].

On the other hand, the prostate stroma invasion by urothelial carcinoma was confirmed in 5 cases (5/34, 14.7%) and one of them had a prostate apex involvement, which was lower than most of the recent reports. In a large series from Pettus et al, 39 out of 122 patients (32%) were found to have prostatic urothelial carcinoma involvement with apical involvement in 18 specimens (15%) [42]. Shen et al also reported a 32% prostate involvement rate with urothelial carcinoma in RCP specimens for bladder cancer [43]. From these studies, we may find that bladder tumor stage, tumor grade, multifocality, tumor in bladder neck/trigone and presence of carcinoma in situ are important risk factors for prostate involvement. Patients with such risk factors are not appropriate candidates for prostate-apex sparing surgery.

Even though the probability of tumor residual in prostate apex is really low, the local recurrence could lead to serious problem in patients with orthotopic neobladder. Therefore, a positive preoperative prostate apical biopsy should preclude the apex-sparing RCP. However, since most incidentally detected prostate cancer are insignificant tumor with a tumor volume<0.5 ml, a negative biopsy cannot completely exclude apical involvement in these patients [44]. Currently no reliable preoperative factors are available to adequately identify whether patients with prostate cancer in the apex [45]. Meanwhile, considering the possibility of concomitant invasion of prostate apex by urothelial carcinoma, we believe the inclusion criteria for prostate apex-sparing surgery in Chinese patients should be limited as follows: young age (<60 years) and socially active, normal erectile function, normal DRE, pT2 solitary bladder cancer, no urothelial carcinoma in trigone, in bladder neck or in prostatic urethra and without carcinoma in situ. Hence, as the preoperative workup, an erectile function assessment before the surgery, a DRE, a serum PSA examination, a pelvic MRI and a cystoscopy with randomized biopsy should be absolutely essential in order to carefully evaluate these candidates.

Besides the apex-sparing radical cystoprostatectomy, there are other techniques such as prostate sparing cystectomy and bladder sparing strategies offering patients better quality of life when treating the muscle invasive bladder cancer. Theoretically, whole prostate sparing cystectomy might have more risk of leaving prostate cancer or urothelial carcinoma in prostate. A Canadian study revealed the overall rate of an underlying cancer within the prostate of cystoprostatectomy specimens was about 46% [46]. Mertens et al reported a 20-year single center experience of prostate sparing cystectomy for bladder cancer with a satisfactory oncological outcome [47]. The 2 and 5-year recurrence-free survival rates were 71.2% and 66.6% with complete daytime and nighttime continence in 96.2% and 81.9% of patients and erectile function intact in 89.7% of patients. Since the whole prostate was preserved, the patient selection should be very careful before the surgery. In their study, all patients underwent preoperative transurethral biopsy of the bladder neck and prostatic urethra and transrectal biopsies of prostate to rule out tumor in the bladder neck, prostatic urethra or prostate cancer. Meanwhile, the bladder sparing strategy is also a feasible procedure in well selected cases. Coen et al carried out a study of 325 cases with muscle invasive bladder cancer treated by transurethral resection and chemoradiation [48]. They established a nomogram including information on clinical T stage, presence of hydronephrosis, whether a visibly complete transurethral resection of bladder tumor was performed, age, sex, and tumor grade to predicting response to bladder-sparing therapy and oncological outcomes. Zapatero et al reported the long-term outcome of prospective bladder-sparing trimodality approach for invasive bladder cancer [49]. Five and 10-year cumulative overall survival were 60%–73% and the cancer-specific survival was 80%–82%. Of all surviving patients, 83% maintained their own bladder. However, these studies of bladder-sparing approach didn't report the erectile function of the patients after chemotherapy and radiotherapy while the chemoradiation could have great influence on it.

Limitation of our study was its retrospective nature. In this study, of all the 504 cases enrolled, the preoperative PSA was only available in 296 cases before radical cystoprostatectomy. For the rest of 208 cases without preoperative PSA, even no palpable nodule was found by DRE, the patients could have concomitant clinical prostate cancer which hadn't been discovered before the surgery. This might lead to a potential selection bias and influence the incidence of incidental prostate cancer in radical cystoprostatectomy specimens, although such an influence could be very limited because of the low incidence of clinical prostate cancer in China (12.10/100 000).A prospective randomized study with large case volumes should be carried out in the near future to evaluate the functional outcome and especially the oncological risk of prostate apex-sparing surgery for bladder urothelial carcinoma in Asia patients.

## Conclusion

The prevalence of incidental prostate cancer in RCP specimens in Chinese patients was remarkably lower than in western people. Most of the incidental prostate cancer was clinically insignificant and the patient's prognosis was mainly related to the bladder cancer. Sparing the prostate apex was potentially associated with a 1.0% risk of leaving significant cancer of the prostate or urothelial carcinoma. Further prospective randomized study with large case volumes should be carried out to evaluate the functional outcome and especially the oncological risk of this technique in Asian patients.
